The article "Automatic Surgery and Anesthesia Emergence Duration Prediction Using Artificial Neural Networks" was published in 2022. Journal: J Healthc Eng.

# Automatic Surgery and Anesthesia Emergence Duration Prediction Using Artificial Neural Networks

**DOI:** 10.1155/2022/2921775

**Published:** 2022-04-14

**Authors:** Li Huang, Xiaomin Chen, Wenzhi Liu, Po-Chou Shih, Jiaxin Bao

**Affiliations:** ^1^Economics and Management School, Panzhihua University, Panzhihua 617000, China; ^2^Business School, University of Shanghai for Science and Technology, Shanghai 200093, China; ^3^Affiliated Hospital, Panzhihua University, Panzhihua 617000, China; ^4^Department of Industrial Engineering and Management, Chaoyang University of Technology, Taichung 413310, Taiwan

## Abstract

Cost control is becoming increasingly important in hospital management. Hospital operating rooms have high resource consumption because they are a major part of a hospital. Thus, the optimal use of operating rooms can lead to high resource savings. However, because of the uncertainty of the operation procedures, it is difficult to arrange for the use of operating rooms in advance. In general, the durations of both surgery and anesthesia emergence determine the time requirements of operating rooms, and these durations are difficult to predict. In this study, we used an artiﬁcial neural network to construct a surgery and anesthesia emergence duration-prediction system. We propose an intelligent data preprocessing algorithm to balance and enhance the training dataset automatically. The experimental results indicate that the prediction accuracies of the proposed serial prediction systems are acceptable in comparison to separate systems.

## 1. Introduction

In recent years, cost savings have become critical in hospitals [1–3]. In addition to staff salaries, hospitals have to pay for equipment, materials, and administrative expenses. A conservative estimate of operating room utilization costs exceeded $15 per minute in 2012 [1]. However, in 2017, the estimate increased to $36 per minute [2]. The cost has always been an important optimization objective in operating room scheduling [3]. Therefore, cost control is a key factor for successful hospital management.

The operating room is a core component of the hospital, and its use contributes considerably to hospital costs [4]. In general, surgeries require expensive resources, such as equipment, materials, energy, and medical staff [5]. In some hospitals, several operating rooms form a laminar flow operation center, in which the energy cost of using five operating rooms for one hour is almost the same as that of using one operating room for one hour. However, the energy cost of using one operating room for five hours is five times that of using five operating rooms for one hour. If the operating rooms are not optimally used, the cost is high. Hence, detailed operating room scheduling is required to ensure that all required resources are available at the right time.

Therefore, a well-arranged operating room schedule can reduce costs. However, such a schedule is difficult to achieve, primarily because of the uncertainty in the operating room use duration [6], which is determined by surgery and anesthesia emergence durations. Surgery duration is defined as the time from the beginning to the end of surgery. Anesthesia emergence duration is the time from the end of the surgery to the time when the patient wakes up. Anesthesia emergence is relevant only in surgeries under general anesthesia. If the operating room schedule does not allocate sufficient time for an operation, the next operation cannot start on time. However, if the planned operation duration is longer than the actual duration, the operating room will be vacant, leading to a waste of resources. In extreme cases, operating rooms may remain open beyond their planned working hours, incurring costly overtime wages and energy consumption [7]. Similarly, an inaccurate estimate of the duration of anesthesia emergence can lead to poor surgical scheduling, resulting in resources wastage. In contrast, optimal scheduling can reduce the resource consumption that is caused by the difference between the estimated and the actual operating room use times.

Previous studies have used several approaches to estimate surgery duration [8–17]. A common method is to assume the decisions of surgeons as the deciding factor. Surgeons make a rough estimate of the operating room use times based on the average duration of previous similar operations (previous experience), the type of surgery, patient characteristics, and other factors. [8]. They tend to avoid risks and have limited ability to estimate the duration of surgery [9]. Using this method, the case duration was overestimated by up to 32% or underestimated by 42% [10]. The second common approach is to use electronic health records (EHRs) to calculate a given case duration based on historical data [11]. Because EHR does not take into consideration factors, such as body mass index, anesthesia type, staff, and so on [12], its accuracy is modestly higher for ordinary patients [11] and greatly dependent on other factors. Another method is to simulate the case duration according to the concept of probability distribution. Commonly used probability distributions include the hypergamma, lognormal, gamma, and Weibull distributions [13]. This approach has often been used to describe the stochastic duration of surgery, however, its accuracy has not been reported in the literature. With the popularization of artificial intelligence, numerous statistical and machine-learning tools have been used to predict surgery durations. These methods include Bayesian methods [14], regression techniques [14–16], neural networks [14–16], and random forests [17]. For example, Devi et al. [14] established neural networks and regression models for three types of ophthalmic surgery studies (cataract, corneal transplant, and oculoplastic surgery). The predicted root mean square error was affected by the number of hidden layer neurons constructed by the model. Because of the different types of surgeries, the RMSE was 0.0656–0.6295. Based on the findings of reference [14], we conducted more in-depth experiments on the decision-making of prediction model architecture, including the number of hidden layers and the number of neurons in each hidden layer.

Bartek et al. [15] used linear regression and supervised machine learning to create surgeon-specific models (92 individual models) and service-specific models (12 service-specific models). The prediction accuracies of the former were 32% to 39% and better than those of the latter. Shahabikargar et al. [17] employed the filtered random forest algorithm to predict the surgical duration. They filtered the data of 60,362 elective surgeries in two hospitals by deleting missing, inconsistent, and duplicate values before modeling. The overall prediction error decreased by 44% (mean absolute percentage error from 0.68 to 0.38%) compared to the error without data preprocessing. Therefore, for data preprocessing, we referred to the data cleaning operation in reference [17] and proposed an intelligent data preprocessing algorithm to improve the data quality.

Tuwatananurak et al. [16] employed supervised learning to learn 990 effective surgical data within three months. The results showed a 7 min improvement in absolute difference between the predicted and actual case durations when compared to that obtained using conventional EHR. The method also resulted in a 70% reduction in overall scheduling inaccuracy. As hospitals seek more economical process arrangements, the patient's anesthesia recovery is being moved from the operating room to the postanesthesia care unit, resulting in the separation of anesthesia recovery time from operation time. Thus, these two must be predicted separately. To the best of our knowledge, no study has been reported on the prediction of anesthesia awakening time. Therefore, in this study, we constructed a serial artificial neural network (ANN) to predict the operation and anesthesia recovery time.

Artificial intelligence has been recently adopted to various prediction problems and has resulted in good prediction performance. For example, an ANN was used to predict the recidivism of commuted prisoners [18] and solve the ship detection problem [19]. A support vector machine (SVM) was used to classify the reclaimed wafers into good and not good categories [20]. The driver lane-keeping ability in the fog problem was solved using an association rule [21]. The ANN has been used to solve various types of prediction problems and has better accuracy than SVM in supervised learning [20, 22]. Therefore, to predict the duration of surgery and anesthesia emergence more accurately for arranging the operating rooms more efficiently and effectively, ANN was used to construct the surgery duration prediction system in our previous study [23], and we used ANN to construct the anesthesia emergence duration prediction system in this study. The anesthesia emergence duration is affected by the surgery duration: the longer the surgery duration, the longer the anesthesia emergence duration. Thus, the former is an input variable for the anesthesia emergence duration prediction system. However, the actual surgery duration is unknown before the procedure is performed. Therefore, we, firstly, constructed two prediction systems: surgery duration and anesthesia emergence duration prediction systems, and then combined them to obtain the final prediction system. We used the predicted surgery duration as the input variable for the anesthesia emergence duration prediction system. According to the experimental results, the prediction accuracy of the final prediction system was 95.52%. Besides, we developed an intelligent data preprocessing algorithm to balance and enhance the dataset for the ANN. This algorithm automatically calculates the most appropriate replication time.

The remainder of this paper is organized as follows: Section 2 introduces the ANN, perceptron, and multilayer perceptron (MLP).  Section 3 describes the experiments conducted and the data preprocessing algorithm.  Section 4 discusses the experimental results of the three prediction systems: surgery duration, anesthesia emergence duration, and final prediction systems. Finally, the conclusions and suggestions for future research are presented in Section 5.

## 2. Review of the Artificial Neural Network

### 2.1. Artificial Neural Network

An ANN is a complex artificial system based on mathematical models based on the function, structure, and information processing of the human brain and nervous system [24, 25]. Similar to the human brain, an ANN is a self-learning system that learns to predict outputs by performing numerous iterations. All types of ANN nodes are akin to the neurons in the human brain, each of which is used as the input of the next node, after the weighting function [26, 27]. In the learning process, the weights are updated using a systematic algorithm. To obtain better output accuracy, the ANN often performs the backpropagation learning algorithm, i.e., it uses a certain set of weights and biases to perform an iteration, calculate the error with the output and actual value, propagate backwards, and update the weights and bias by the error to ensure that after several such forward and backward propagations, the output accuracy is high [28, 29]. After the ANN is trained, new data can be classified or predicted using the received stimulus (new input data), weights, and biases.

The ANN is a powerful tool for learning and modeling complex linear or nonlinear relationships. To be more precise, the model it builds is similar to a “black box.” The nature of the relationship between the input and output data is unknown [30]. ANNs have been widely applied in a wide range of problems in multiple fields, including engineering [31, 32], biology, mathematics, and medicine, to analyze and predict various diseases [33].

### 2.2. Perceptron

The perceptron model was derived from the MP model established by McCulloch and Pitts [34]. By simulating the principles and processes of biological nerve cells, the MP model describes the mathematical theory and network structure of artificial neurons and proves that a single neuron can realize a logical function. The MP model contains input, output, and computation functions. The input and output are analogous to the dendrite and axon of a neuron, respectively, whereas the calculation is similar to the processing conducted in the nucleus, with each synapse being assigned a weight.

Inspired by the MP model, the perceptron model consists of two layers. The first layer, called the input layer, receives the stimulus and passes it to the last layer. In the final layer, called the output layer, all input stimuli are multiplied with their respective weights, and the perceptron adds all the weighted stimuli and bias using the summation function. Finally, the perceptron uses an activation function to simulate data processing in the brain [35]. The basic network structure of a perceptron is shown in Figure 1.

### 2.3. Multilayer Perceptron

To better handle nonlinear problems, Hecht-Nielsen proposed a multilayer perceptron by placing additional layers (s) of neurons between the input and output layers [35]. As shown in Figure 2, there are two fundamental components of the basic MLP structure: neurons and the links between neurons. The *n*_*i*_ neurons are the processing elements, and the links are interconnections. Every link has a corresponding weight parameter *w*_*j*_ or bias parameter *b*_*i*_. When a neuron receives stimuli from other neurons via links, it processes the information and produces an output. Moreover, these intermediate layers are assumed to not be disturbed by the external environment. Therefore, they are called hidden layers, and the nodes of hidden layers are called hidden nodes. Similar to the perceptron, the input neurons receive external stimuli, and the output neurons deliver the output. Using similar neuron dynamics, hidden neurons receive stimuli from neurons at the front of the network and relay the output to the neurons at the back of the network [18].

## 3. Experiments

### 3.1. Data Setting

Operational records collected between January 2019 and July 2020 from the Affiliated Hospital of Panzhihua University were used as samples in this study. The records were used only for academic purposes and were anonymized to protect privacy.

In total, 15,754 samples were collected for this study. These samples were the data of patients without hepatic and renal diseases. To eliminate potential factors that could influence the operation time, all samples from emergency surgery patients or patients admitted to the intensive care unit after surgery were excluded. Thus, records from only patients with complete case data were included. Samples with all types of anesthesia were considered to predict the duration of surgery, whereas only samples under general anesthesia were considered to predict the duration of anesthesia emergence.

To improve the prediction accuracy of the model, we collected the data available preoperatively and identified the influencing factors of surgery and anesthesia emergence durations as the input variables of the model through literature survey and physician interviews. The input and output variables of the surgery and anesthesia emergence duration prediction systems are presented in Tables 1 and 2, respectively. In Table 1, the input variables are composed of three parts: basic patient information and preoperative physiological data (A1–A18), surgeon information (A20–A23), and operation information (A19 and A24). In Table 2, the input variables are composed of three parts: basic patient information and preoperative physiological data (A1–A18), anesthesiologist information (A20–A23), and operation information (A19 and A24). By comparing these tables, we observed that the 20^th^ and 24^th^ input variables of the two systems were different. Firstly, as mentioned in the data setting criteria, samples with both local and general anesthesia were used in the first system, whereas only samples with general anesthesia were used in the second system. Hence, they were subdivided into four types of general anesthesia. Furthermore, the duration of surgery was dependent on the surgeon, whereas the duration of anesthesia emergence was dependent on the anesthesiologist. Moreover, the surgical grade had a profound impact on the duration of surgery but a negligible effect on the duration of anesthesia emergence. Hence, it was ignored in the latter case. In summary, the duration of surgery may affect the duration of anesthesia emergence. Therefore, the output variable of the first system was used as the 24th input variable of the second system. Given that the duration of surgery was less than 4 h, all samples with a duration of less than 4 h were used to predict the duration of surgery. Given that most durations of anesthesia emergence are less than 1 h, all samples with a duration of less than 1 h were used to predict the duration of anesthesia emergence. Therefore, the last row of Table 1 shows that the surgery duration was divided into four scales: no more than one hour, 1 h to 2 h, 2 h to 3 h, and 3 h to 4 h. Similarly, the duration of anesthesia emergence was divided into four scales: no more than 15, 15 to 40, 40 to 50, and 50 to 60 min, as shown in the last row of Table 2.

The success of an ANN depends heavily on appropriate data preprocessing. Hence, all data in this study were preprocessed using data transformation [36], inspection [37], and exclusion of outliers. After data preprocessing, 6,507 and 5,790 surgery samples were retrospectively used to predict the durations of surgery and anesthesia emergence, respectively. In addition, normalizing the data is recommended to avoid gradient explosion and eliminate the influence of data heterogeneity, which can hinder the learning process [38]. All the data normalized ranged between 0.1 and 0.9. Moreover, balancing and enriching data are essential steps in solving classification problems [39]. We propose an intelligent data-preprocessing algorithm to balance and enhance the dataset. Thereafter, we divided the dataset into training, testing, and validation datasets. The most important process of this algorithm was data balancing. The purpose of data balancing is to reduce the differences in the amount of data in each category. Two examples of data balancing are shown in Figure 3. *n*_*i*_ indicates the amount of data in category *i*, and *n*_max_ indicates the maximum of *n*_*i*_. All categories must balance the data based on *n*_max_. In Figure 3, for example, *n*_1_ represents the amount of data in Category 1 and is equal to 60. *n*_max_ is equal to 100. Category 1 must balance data based on *n*_max_. The difference between the original *n*_1_ (60) and *n*_max_ (100) values is 40. If we increase the amount of data in categories 1 to 120, the difference between 2 × *n*_1_ (120) and *n*_max_ (100) decreases to 20. Therefore, in category 1, the best multiple was 2. In another example, *n*_2_ indicates the amount of data in category 2 and is equal to 30. If we increase the amount of data in categories 2 to 90, the difference between 3 × *n*_2_ (90) and *n*_max_ (100) is 10. However, if the amount of data in categories 2 to 120 is increased, the difference between 4 × *n*_2_ (120) and *n*_max_ (100) increases to 20. Therefore, in category 2, the best multiple is 3. Based on the above concept, the rules of multiplication for data balancing are listed in Table 3. In Table 3, if 2/*k* − 2*n*_max_ ≥ *n*_*i*_ > 2/*kn*_max_, the multiple of the data balance is *k* − 1/2. The main process of the intelligent data preprocessing algorithm is illustrated in Figure 4. This algorithm requires only the normalized data, multiple to be used for enhancement, and the partition ratio of the dataset as input. Finally, we obtained the balanced, enhanced, and partitioned dataset. We generated new samples and expanded the database size by adding slight noise to the input data while maintaining the same output category. The value of the noise was between −0.03 and +0.03.

After data balancing, the data were increased by three times in the initial experiments and ten times in the final experiment. In addition, data representation was an essential part of a successful ANN [37]. In this study, the output variable was categorized according to four binary numbers, namely, 1000, 0100, 0010, and 0001, where the position of 1 indicates the category.

### 3.2. Computing Environment Settings

We used Python 3.7 (64 bit) as the compiler to write the program. The hardware included an Intel Core (TM) i7-10510U (2.3 GHz) CPU, 8 GB of memory, and Windows 10 Home Edition (64 bit) operating system.

### 3.3. Experimental Structure

The experiment was conducted in two parts. In the first part, we used MLP to construct the surgery duration prediction system and the anesthesia emergence duration prediction system. To determine the optimal architecture of both models, we conducted two sets of experiments with the same data partitioning and parameter settings. The total dataset was divided into three datasets, namely training, testing, and validation, in the respective proportions of 60, 20, and 20% [39, 40].

In the MLP, the Adam optimizer was used to adjust the weights and the cross-entropy loss function to calculate the loss of the prediction system. The batch size was set to 100, and the number of training cycles was set to 200 and 1,000 in the final experiment of the optimal architecture. The number of hidden layers and hidden nodes in each layer are critical determiners of the results [35, 39, 41]. We used a trial-and-error method to identify an optimal number of hidden layers and hidden nodes. The number of hidden layers was set to three, four, five, and six, and the number of hidden layer nodes of each layer was set to 64, 128, 256, and 512, respectively. Thus, the experimental results of the 16 parameter combinations were obtained for comparison and analysis. To reduce the stochastic effects of the experiments, we conducted ten experiments for each parameter combination. Finally, we obtained the two optimal architectures and weights used in the second part. Figures 5 and 6 show the MLP structure of the surgery duration prediction system and anesthesia emergence duration prediction system, respectively.

In the first part, we used the actual duration of surgery as the input variable of the second model. However, as mentioned in Section 3.1, the output variable of the first model was the input variable of the second model. Therefore, in the second part, we merged these two prediction systems into one. In other words, we used the predicted duration of surgery as an input variable for the second model. Thus, we intersected 6,507 surgery samples with 5,790 anesthesia emergence prediction samples and obtained 4,285 samples. The predicted surgical duration was obtained by feeding the samples into the first prediction system. The predicted duration of surgery was combined with other attributes of the samples and fed into the second prediction system to determine the duration of anesthesia emergence.  Figure 7 shows the final combination prediction system.

## 4. Experimental Results and Analysis

### 4.1. Experimental Results of the Surgery Duration Prediction System

We used a trial-and-error method to identify the final architecture of the surgery duration prediction system. The experimental results are listed in Tables 4–11. Tables 4 and 5 present the prediction accuracy and loss value, respectively, of the surgery duration prediction system. In addition, to further explore the performance of several different MLP architectures, the experimental results were analyzed using the *t*-test, as shown in Tables 6–10.  Table 11 lists the running time costs for each architecture. We determined the final architecture of the MLP based on the maximum prediction accuracy and a reasonable running time cost.

In Table 4, **Mean** and **Std** indicate the average prediction accuracy and standard deviation, respectively, over ten experiments. **Max** and **Min** indicate the maximum and minimum prediction accuracies during 10 experiments, respectively. Here, 3-64 denotes the MLP model with 3 hidden layers and 64 hidden neurons in each hidden layer. In the three hidden layer architectures in Tables 4 and 5, the 3-512 architecture had the maximum average prediction accuracy (0.7254) and the minimum loss value (0.6664) in the testing dataset. As shown in Table 6, the 3-512 architecture is significantly better than the 3-64 and 3-128 architecture. However, the 3-512 architecture is not significantly better than the 3-256 architecture. The *p* value is 0.4854. In other words, the 3-512 architecture and 3-256 architecture had similar prediction accuracies. In Table 11, we notice that the 3-512 architecture had a longer running time (1806.50 s) than the 3-256 architecture (584.24 s). In other words, among the three hidden layer architectures, the 3-256 architecture reduced runtime costs by 67.66% compared with the 3-512 architecture. Therefore, in the three hidden layer architectures, we chose the 3-256 architecture prediction system.

In the four, five, and six hidden layer architectures, in Tables 4 and 5, we note that the 4-256, 5-256, and 6-256 architectures had the maximum average prediction accuracies (0.7711, 0.7601, and 0.7493, respectively) and the minimum loss values (0.6551, 0.6579, and 0.6606, respectively) in the testing dataset. In Tables 7 and 8, the MLP model with 256 neurons is significantly better than those with 64 and 128 neurons. However, the MLP model with 256 neurons was not significantly better than the model with 512 neurons. The *p* values were 0.1291 and 0.4207, respectively. In other words, in four-and five-hidden-layer architectures, the MLP models with 256 and 512 neurons had similar prediction accuracies. However, from Table 11, we note that the 4-256 and 5-256 architectures reduced runtime costs by 69.49 and 72.23% compared with the 4-512 and 5-512 architectures, respectively. Therefore, in four and five hidden layer architectures, we chose the 4-256 and 5-256 architecture prediction systems. In Table 9, among the six hidden layer architectures, the 6-256 architecture was significantly better than the other architectures.

In all architectures, in Tables 4 and 5, the 4-256 architecture had the maximum average (**Mean**) prediction accuracies (0.7711, 0.8468, and 0.7714) and the minimum loss values (0.6551, 0.6364, and 0.6550) in the testing, training, and validation datasets, respectively. In addition, the 4-256 architecture had the best maximum (**Max**) and minimum (**Min**) prediction accuracy in almost all the testing, training, and verification datasets. In Table 10, the 4-256 architecture was significantly better than the 3-256 and 6-256 architectures but not significantly better than the 5-256 architecture. However, the *p* value (0.0710) was close to 0.05. In other words, the 4–256 architecture was significantly better than the 5-256 architecture. In addition, in Table 11, the 4-256 architecture saved 18.07% of the runtime cost compared to the 5-256 architecture. Therefore, the final architecture of the surgery duration prediction system is a 4-256 architecture.

After determining the best architecture of the surgery duration prediction system, we further improved the prediction accuracy through dropout mechanism, data enrichment, and longer training time. The experimental results are listed in Tables 12–15. Tables 12 and 13 present the effect of the dropout mechanism, and Tables 14 and 15 present the impact of the data enrichment and longer training time on the 4-256 architecture, respectively. In Tables 12 and 13, we note that the 4-256 architecture without the dropout mechanism had the maximum average prediction accuracy (0.7711) and minimum loss value (0.6551) in the testing dataset. With an increase in the dropout probability, the average prediction accuracy decreases. In other words, the dropout mechanism cannot improve the prediction accuracy of the surgery duration prediction system. We enriched the data 10 times, and in Tables 14 and 15, the 4-256 architecture with 10 times the data had a better average prediction accuracy (0.8788) and loss value (0.6284) in the testing dataset. We also increased the training time to 1,000 epochs and found that the average prediction accuracy increased to 0.9485, and the average loss value decreased to 0.6110 in the testing dataset. In other words, data enrichment and increasing training time improved the prediction accuracy of surgery duration prediction system. The final architecture of the surgery duration prediction system is the 4-256 architecture without dropout mechanism, trained with 10 times the data over 1,000 epochs.

### 4.2. Experimental Results of the Anesthesia Emergence Duration Prediction System

We used a trial-and-error method to determine the final architecture of the anesthesia emergence duration prediction system. The experimental results are presented in Tables 16–23. Tables 16 and 17 present the prediction accuracy and loss values of the model, respectively. To further explore the performance of several different MLP architectures, the experimental results were also analyzed using *t*-tests, as shown in Tables 18–22.  Table 23 lists the running time costs for each architecture. We determined the final architecture of the MLP based on the maximum prediction accuracy and a reasonable running time cost.

In the three hidden layer architectures in Tables 16 and 17, the 3-512 architecture had the maximum average prediction accuracy (0.7391) and the minimum loss value (0.6632) in the testing dataset. As shown in Table 18, the 3-512 architecture was significantly better than the 3-64 and 3-128 architectures. However, the 3-512 architecture is not significantly better than the 3-256 architecture. The *p* value was 0.4726. In other words, the 3-512 architecture and 3-256 architecture had similar prediction accuracies. In Table 23, we note that the 3-512 architecture have a longer running time (1928.91 s) than the 3-256 architecture (613.93 s); hence, the 3-256 architecture reduced the runtime cost by 68.17%. Therefore, we determine that the 3-256 architecture was the best architecture for the prediction system.

In the four and five hidden layer architectures, as listed in Tables 16 and 17, the 4-256 and 5-256 architectures show the maximum average prediction accuracies (0.7836 and 0.7905, respectively) and the minimum loss values (0.6520 and 0.6503, respectively) in the testing dataset. In Table 19, the 4-256 architecture is significantly better than the 4-64 and 4-128 architectures, but not significantly better than the 4-512 architecture. However, the *p* value (0.0892) was close to 0.05. In other words, the 4-256 architecture was significantly better than the 4-512 architecture. In Table 23, the 4-256 architecture saved 68.15% of the runtime cost compared with the 4-512 architecture. Therefore, among the four hidden layer architectures, we determine that the best architecture of the prediction system was the 4-256 architecture. In Table 20, the 5-256 architecture is significantly better than the other five hidden-layer architectures.

In the six hidden layer architectures, in Tables 16 and 17, the 6-128 architecture have the maximum average prediction accuracy (0.7454) and the minimum loss value (0.6616) in the testing dataset. As shown in Table 21, the 6-128 architecture is significantly better than the 6-64 and 6-512 architectures. However, the 6-128 architecture is not significantly better than the 6-256 architecture. The *p* value was 0.3675. Therefore, the 6-128 and 6-256 architectures have similar prediction accuracies. However, as shown in Table 23, the 6-256 architecture have a longer running time (1204.03 s) than the 6-128 architecture (988.21 s). Therefore, the 6-128 reduced the runtime cost by 17.93% and was the best architecture for the prediction system.

In all architectures, as listed in Tables 16 and 17, the 5-256 architecture had the maximum average (**Mean**) prediction accuracies (0.7905, 0.8443, and 0.7924) and minimum loss values (0.6503, 0.6370, and 0.6499) in the testing, training, and validation datasets, respectively. In addition, the 5-256 architecture had the best maximum (**Max**) and minimum (**Min**) prediction accuracy in almost all testing, training, and verification datasets. In Table 22, the 5-256 architecture was significantly better than the 3-256 and 6-128 architectures, but not significantly better than the 4-256 architecture. The 5-256 architecture and 4-256 architecture have similar prediction accuracies. Finally, in Table 23, the 4-256 architecture reduced the runtime costs by 26.90% compared to the 5-256 architecture. Therefore, we determine that the final architecture of the anesthesia emergence duration prediction system is the 4-256 architecture.

After we determined the best architecture of the anesthesia emergence duration prediction system, we further improved the prediction accuracy using the dropout mechanism, data enrichment, and longer training time. The experimental results are listed in Tables 24–27. Tables 24 and 25 present the effect of the dropout mechanism, and Tables 26 and 27 present the impact of data enrichment and longer training time on the 4-256 architecture. In Tables 24 and 25, we can easily observe that the 4-256 architecture without the dropout mechanism had the maximum average prediction accuracy (0.7836) and minimum loss value (0.6520) in the testing dataset. With an increase in dropout probability, the average prediction accuracy decreases. Thus, the dropout mechanism cannot improve the prediction accuracy of the anesthesia emergence duration prediction system. We then enriched the data ten times. In Tables 26 and 27, the 4-256 architecture with 10 datasets had a better average prediction accuracy (0.8956) and loss value (0.6242) in the testing dataset. We increased the training time to 1,000 epochs, and we determined that the average prediction accuracy increased to 0.9544, and the average loss value decreased to 0.6095 in the testing dataset. Finally, the architecture of the anesthesia emergence duration prediction system is a 4-256 architecture without a dropout mechanism, trained with 10 times of data over 1,000 epochs.

### 4.3. Experimental Results of the Final Combination Prediction System

In this section, we discuss the results of the final system obtained by combining the surgery duration prediction system with the anesthesia emergence duration prediction system. As mentioned in Section 1, we predicted the duration of anesthesia emergence using the surgery duration. However, we could not obtain the actual duration before surgery. We then used the predicted surgery duration as the input variable for the anesthesia emergence duration prediction system. As mentioned in Section 3.3, we used 4,285 samples in the final combination prediction system. To compare the prediction accuracy of the final combination prediction system, we used 4,285 samples in the surgery duration prediction system and the anesthesia emergence duration prediction system. The experimental results are listed in Table 28.

As shown in Table 28, the prediction accuracy of the anesthesia emergence duration prediction system is 0.9645. It means that 96.45% of the anesthesia emergence duration prediction accuracy can be obtained by inputting the actual surgery duration. The prediction accuracy of the surgery duration prediction system is 0.9671. It indicates that in the final combination prediction system, the input variable A_24_ is 96.71% correct. Finally, the prediction accuracy of the final combination prediction system is 0.9645. It implies that 95.52% of the anesthesia emergence duration prediction accuracy can be obtained by inputting 96.71% of the correct prediction of surgery duration time. This value (95.52%) was close to 96.45%. The difference between these two prediction systems is only 0.93% and less than 1%. Thus, the prediction accuracy of the final combination prediction system is acceptable.

## 5. Conclusion and Future Research

In this study, we proposed an intelligent data preprocessing algorithm that balances data automatically and used the MLP model to construct the surgery and anesthesia emergence duration prediction systems. Based on existing patient data, we identified the main attributes that affected the prediction of surgery duration and anesthesia emergence duration and then preprocessed the data accordingly. These two systems were extensively tested, compared, and analyzed to determine their implementation. By combining these two prediction systems, we were able to predict the duration of anesthesia emergence from the predicted duration of surgery. There are several interesting findings from the experimental results.

Firstly, the proposed intelligent data preprocessing algorithm has three functions: data balance, data enhancement, and dataset partitioning. In particular, it can calculate the proper multiples of each category to balance the data automatically, depending on the amount of data in each category. Using this algorithm, we did not need to calculate the multiples for each category. Therefore, our workload on data balancing was reduced, especially for a large number of categories. No similar automatic processing algorithm has been found in the limited literature research. Therefore, we thought that the proposed algorithm could be extended to the data balance of data preprocessing. Secondly, the model architecture parameters have an important impact on the prediction accuracy of the model, which is consistent with the research findings of literature [14]. In their study, they took ophthalmic surgery as the research object and found that the prediction error of the model was affected by the number of hidden layer neurons. In our research, we further expanded the exploration of the model architecture and found that 4–256 architecture is the most suitable for both prediction systems. Besides, we found that the smaller the architecture, the lower the accuracy. Conversely, the larger the architecture, the longer the running time. It also shows the importance and necessity of exploring model architecture parameters. Thirdly, overtraining did not occur. Therefore, the dropout mechanism could not improve the prediction accuracy of the two prediction systems. However, data augmentation and longer learning period improved the prediction system. These results are consistent with the theory of artificial neural network. In addition, in literature [16, 17], the influence of data quality on the prediction accuracy of the model was studied, and it was found that data quality affects the prediction accuracy of the model. In this study, we found that the quantity and quality of data are very important to the prediction accuracy of the model. Finally, before the operation is performed, it is very important to predict the surgery and anesthesia emergence duration in advance for the effective scheduling of the operation. Therefore, after combining these two prediction systems, we used the predicted surgery duration to accurately predict the anesthesia emergence duration. Based on the prediction accuracy, the combination of these two prediction systems is acceptable.

It is worth noting that the data used in this study were collected from the Affiliated Hospital of Panzhihua University in China. Therefore, one of the limitations of this study is that the experimental results of this study may only be applicable to the same type of hospitals in China. Besides, we still have many variables that were not considered in this study, such as the data for physical examination before surgery. In fact, we attempted to collect preoperative physical examination data and integrate them with the data used in this study. However, we found too many missing values in the physical examination data. We hypothesize that the main reason for this is that patients undergo different physical examinations. Therefore, the integrated data contained a large number of missing values. We also believe that patients undergoing the same type of surgery should undergo the same physical examination. Therefore, we suggest that in the future, depending on the organs that are subject to surgery, we could use specific physical examination items to predict the surgery duration and anesthesia emergence duration and obtain a more accurate prediction system. Finally, we aimed to predict the exact duration of surgery and anesthesia emergence duration. It can enable the scheduling of surgery to achieve resource use optimization, energy saving, carbon reduction, cost savings, and improve patient's satisfaction. If we can accurately predict the actual surgery time, we will be able to optimize the surgery schedule. However, in practice, there are too many uncertain factors that will affect the prediction of surgery time, which makes it difficult to accurately predict the actual surgery time. Therefore, in our study, we converted the actual surgery time into a time interval (1 hour) to improve the accuracy of prediction. However, if the length of the time interval is too long, it will affect the optimization of surgical scheduling. Therefore, in the future, we suggest that the length of the time interval could be shortened, e.g., to 30 minutes, to improve the optimization of surgical scheduling. Besides, in the future, we also intend to use the predicted surgery and anesthesia emergence durations to further research operating room scheduling.

## Figures and Tables

**Figure 1:** Basic structure of perceptron.

**Figure 2:** Basic structure of MLP.

**Figure 3:** Two examples of data balancing.

**Figure 4:** Intelligent data preprocessing algorithm flow chart.

**Figure 5:** MLP structure to predict duration of surgery.

**Figure 6:** MLP structure to predict duration of anesthesia emergence.

**Figure 7:** Final combination prediction system.

**Table 1:** Input and output variables of the surgery duration prediction system.

Variables	Name	Description
Input	1. Gender (*A*_1_)	(1) Male
		(2) Female
	2. BMI (*A*_2_)	Body mass index
	3. SBP (*A*_3_)	Systolic blood pressure
	4. DBP (*A*_4_)	Diastolic blood pressure
	5. PR (*A*_5_)	Pulse rate
	6. RR (*A*_6_)	Respiration rate
	7. Temperature (*A*_7_)	Body temperature
	8. Heart function classification (*A*_8_)	(1) I level
		(2) II level
		(3) III level
	9. RBC (*A*_9_)	Red blood cell
	10. HB (*A*_10_)	Hemoglobin
	11. HCT (*A*_11_)	Hematocrit
	12. PLT (*A*_12_)	Platelet
	13. K (*A*_13_)	Potassium
	14. NA (*A*_14_)	Sodium
	15. CL (*A*_15_)	Chlorine
	16. APTT (*A*_16_)	Activated partial thromboplastic time
	17. PT (*A*_17_)	Prothrombin time
	18. TT (*A*_18_)	Thrombin time
	19. American society of anesthesiologists (ASA) classification (*A*_19_)	(1) I level
		(2) II level
		(3) III level
	20. Anesthesia type (*A*_20_)	(1) Local anesthesia
		(2) General anesthesia
	21. Surgeon title (*A*_21_)	(1) Physician
		(2) Attending physician
		(3) Deputy chief physician
		(4) Chief physician
	22. Seniority of surgeon (*A*_22_)	The working years of surgeon
	23. Age of surgeon (*A*_23_)	—
	24. Surgical grade (*A*_24_)	(1) Small
		(2) Medium
		(3) Large
		(4) Super
Output (original)	Duration of surgery (*T*)	(1) ≤1 hour
		(2) 1-2 hours
		(3) 2-3 hours
		(4) 3-4 hours
Output (statistical)	Duration of surgery (*T*)	(1) 1000
		(2) 0100
		(3) 0010
		(4) 0001

**Table 2:** Input and output variables of the anesthesia emergence duration prediction system.

Variables	Name	Description
Input	1. Gender (*A*_1_)	(1) Male
		(2) Female
	2. BMI (*A*_2_)	Body mass index
	3. SBP (*A*_3_)	Systolic blood pressure
	4. DBP (*A*_4_)	Diastolic blood pressure
	5. PR (*A*_5_)	Pulse rate
	6. RR (*A*_6_)	Respiration rate
	7. Temperature (*A*_7_)	Body temperature
	8. Heart function classification (*A*_8_)	(1) I level
		(2) II level
		(3) III level
	9. RBC (*A*_9_)	Red blood cell
	10. HB (*A*_10_)	Hemoglobin
	11. HCT (*A*_11_)	Hematocrit
	12. PLT (*A*_12_)	Platelet
	13. K (*A*_13_)	Potassium
	14. NA (*A*_14_)	Sodium
	15. CL (*A*_15_)	Chlorine
	16. APTT (*A*_16_)	Activated partial thromboplastic time
	17. PT (*A*_17_)	Prothrombin time
	18. TT (*A*_18_)	Thrombin time
	19. American society of anesthesiologists (ASA) classification (*A*_19_)	(1) I level
		(2) II level
		(3) III level
	20. Anesthesia type (*A*_20_)	(1) Intravenous general anesthesia
		(2) Intravenous-inhalational balanced anesthesia
		(3) General anesthesia with block anesthesia
		(4) General anesthesia with intraspinal anesthesia
	21. Title of anesthesiologist (*A*_21_)	(1) Physician
		(2) Attending physician
		(3) Deputy chief physician
		(4) Chief physician
	22. Seniority of anesthesiologist (*A*_22_)	The working years of anesthesiologist
	23. Age of anesthesiologist (*A*_23_)	—
	24. Duration of surgery (*A*_24_)	(1) ≤1 hour
		(2) 1-2 hours
		(3) 2-3 hours
		(4) 3-4 hours
Output (original)	Duration of anesthesia emergence (*T*)	(1) ≤15 minutes
		(2) 15–40 minutes
		(3) 40–50 minutes
		(4) 50–60 minutes
Output (statistical)	Duration of anesthesia emergence (*T*)	(1) 1000
		(2) 0100
		(3) 0010
		(4) 0001

**Table 3:** Rules of multiplication on data balancing.

The amount of the data of the category *i* (*n*_*i*_)	The multiple of the data balance
*n*_max_ ≥ *n*_*i*_ > 2*n*_max_/3	(3 − 1)/2=1
2*n*_max_/3 ≥ *n*_*i*_ > 2*n*_max_/5	(5 − 1)/2=2
2*n*_max_/5 ≥ *n*_*i*_ > 2*n*_max_/7	(7 − 1)/2=3
⋮	⋮
2*n*_max_/(*k* − 2) ≥ *n*_*i*_ > 2*n*_max_/*k*	(*k* − 1)/2

**Table 4:** Prediction accuracy of the surgery duration prediction system.

Layers-neurons	Testing dataset				Training dataset				Validation dataset			
	Mean	Std	Max	Min	Mean	Std	Max	Min	Mean	Std	Max	Min
3-64	0.6013	0.0127	0.6173	0.5737	0.6614	0.0140	0.6758	0.6308	0.6033	0.0105	0.6171	0.5789
3-128	0.6830	0.0174	0.6991	0.6374	0.7507	0.0160	0.7656	0.7117	0.6863	0.0122	0.7010	0.6567
3-256	0.7252	0.0131	0.7418	0.7056	0.7996	0.0135	0.8233	0.7797	0.7266	0.0160	0.7556	0.7098
3-512	0.7254	0.0131	0.7491	0.7108	0.7996	0.0117	0.8179	0.7836	0.7261	0.0117	0.7401	0.7093
4-64	0.6506	0.0124	0.6655	0.6260	0.7180	0.0090	0.7305	0.7053	0.6536	0.0115	0.6729	0.6323
4-128	0.7340	0.0118	0.7498	0.7078	0.8084	0.0087	0.8269	0.7955	0.7349	0.0087	0.7564	0.7254
4-256	0.7711	0.0115	0.7919	0.7560	0.8468	0.0118	0.8675	0.8303	0.7714	0.0124	0.7918	0.7564
4-512	0.7639	0.0156	0.7878	0.7312	0.8402	0.0186	0.8681	0.8049	0.7656	0.0161	0.7877	0.7352
5-64	0.6614	0.0111	0.6790	0.6421	0.7335	0.0108	0.7481	0.7139	0.6624	0.0100	0.6771	0.6468
5-128	0.7359	0.0138	0.7582	0.7182	0.8116	0.0129	0.8331	0.7950	0.7329	0.0123	0.7471	0.7165
5-256	0.7601	0.0195	0.7854	0.7272	0.8386	0.0189	0.8608	0.8059	0.7636	0.0182	0.7885	0.7347
5-512	0.7584	0.0168	0.7817	0.7366	0.8365	0.0154	0.8569	0.8140	0.7559	0.0149	0.7848	0.7376
6-64	0.6701	0.0126	0.6916	0.6464	0.7424	0.0158	0.7656	0.7110	0.6680	0.0144	0.6863	0.6368
6-128	0.7201	0.0168	0.7491	0.6948	0.7960	0.0173	0.8269	0.7717	0.7201	0.0158	0.7533	0.7033
6-256	0.7493	0.0161	0.7749	0.7200	0.8297	0.0161	0.8605	0.7994	0.7499	0.0165	0.7740	0.7163
6-512	0.7281	0.0233	0.7548	0.6792	0.8046	0.0234	0.8345	0.7588	0.7271	0.0204	0.7574	0.6858

**Table 5:** Loss value of the surgery duration prediction system.

Layers-neurons	Testing dataset				Training dataset				Validation dataset			
	Mean	Std	Max	Min	Mean	Std	Max	Min	Mean	Std	Max	Min
3-64	0.6974	0.0030	0.7041	0.6936	0.6828	0.0034	0.6903	0.6795	0.6969	0.0026	0.7029	0.6935
3-128	0.6771	0.0042	0.6882	0.6735	0.6604	0.0040	0.6701	0.6567	0.6763	0.0031	0.6839	0.6731
3-256	0.6665	0.0032	0.6712	0.6626	0.6481	0.0033	0.6529	0.6423	0.6662	0.0039	0.6705	0.6590
3-512	0.6664	0.0032	0.6700	0.6605	0.6481	0.0030	0.6521	0.6435	0.6664	0.0030	0.6708	0.6627
4-64	0.6850	0.0028	0.6907	0.6818	0.6686	0.0022	0.6717	0.6656	0.6843	0.0028	0.6891	0.6797
4-128	0.6643	0.0028	0.6703	0.6604	0.6459	0.0022	0.6492	0.6412	0.6641	0.0022	0.6665	0.6587
4-256	0.6551	0.0028	0.6588	0.6501	0.6364	0.0029	0.6404	0.6312	0.6550	0.0030	0.6586	0.6501
4-512	0.6569	0.0038	0.6649	0.6511	0.6380	0.0046	0.6467	0.6311	0.6565	0.0039	0.6639	0.6513
5-64	0.6824	0.0029	0.6876	0.6779	0.6646	0.0027	0.6693	0.6610	0.6821	0.0025	0.6860	0.6785
5-128	0.6639	0.0034	0.6682	0.6583	0.6451	0.0032	0.6492	0.6398	0.6645	0.0031	0.6688	0.6611
5-256	0.6579	0.0048	0.6661	0.6517	0.6383	0.0047	0.6464	0.6327	0.6570	0.0045	0.6640	0.6506
5-512	0.6583	0.0042	0.6639	0.6527	0.6389	0.0038	0.6446	0.6339	0.6589	0.0036	0.6632	0.6519
6-64	0.6802	0.0032	0.6863	0.6748	0.6623	0.0039	0.6702	0.6565	0.6807	0.0036	0.6883	0.6763
6-128	0.6679	0.0043	0.6742	0.6605	0.6489	0.0043	0.6549	0.6413	0.6677	0.0039	0.6719	0.6596
6-256	0.6606	0.0040	0.6680	0.6542	0.6405	0.0040	0.6480	0.6329	0.6604	0.0041	0.6690	0.6544
6-512	0.6659	0.0058	0.6782	0.6595	0.6468	0.0058	0.6581	0.6394	0.6661	0.0050	0.6761	0.6585

**Table 6:** The *t*-test in 3 hidden layer architecture.

Architecture	3-128	3-256	3-512
3-64	0.0000^*∗*^	0.0000^*∗*^	0.0000^*∗*^
3-128	—	0.0000^*∗*^	0.0000^*∗*^
3-256	—	—	0.4854

**Table 7:** The *t*-test in 4 hidden layer architecture.

Architecture	4-128	4-256	4-512
4-64	0.0000^*∗*^	0.0000^*∗*^	0.0000^*∗*^
4-128	—	0.0000^*∗*^	0.0001^*∗*^
4-256	—	—	0.1291

**Table 8:** The *t*-test in 5 hidden layer architecture.

Architecture	5-128	5-256	5-512
5-64	0.0000^*∗*^	0.0000^*∗*^	0.0000^*∗*^
5-128	—	0.0025^*∗*^	0.0021^*∗*^
5-256	—	—	0.4207

**Table 9:** The *t*-test in 6 hidden layer architecture.

Architecture	6-128	6-256	6-512
6-64	0.0000^*∗*^	0.0000^*∗*^	0.0000^*∗*^
6-128	—	0.0004^*∗*^	0.1942
6-256	—	—	0.0145^*∗*^

**Table 10:** The *t*-test in 3–6 hidden layer architectures.

Architecture	4-256	5-256	6-256
3-256	0.0000^*∗*^	0.0001^*∗*^	0.0009^*∗*^
4-256	—	0.0710	0.0013^*∗*^
5-256	—	—	0.0979

**Table 11:** Running time cost of each architecture of the surgery duration prediction system.

Architecture	Time (s)
3-64	339.72
3-128	404.73
3-256	584.24
3-512	1806.50
4-64	375.72
4-128	474.83
4-256	756.63
4-512	2480.10
5-64	404.15
5-128	560.63
5-256	923.48
5-512	3325.30
6-64	448.18
6-128	622.16
6-256	1072.77
6-512	4155.28

**Table 12:** Prediction accuracy of the surgery duration prediction system with dropout mechanism.

Architecture	Dropout	Testing dataset				Training dataset				Validation dataset			
		Mean	Std	Max	Min	Mean	Std	Max	Min	Mean	Std	Max	Min
4-256	**Without**	**0.7711**	0.0115	**0.7919**	**0.7560**	**0.8468**	0.0118	**0.8675**	**0.8303**	**0.7714**	0.0124	**0.7918**	**0.7564**
	0.1	0.7287	0.0115	0.7485	0.7112	0.8112	0.0120	0.8289	0.7907	0.7298	0.0122	0.7466	0.7093
	0.2	0.6562	**0.0058**	0.6648	0.6474	0.7263	**0.0056**	0.7349	0.7178	0.6558	**0.0048**	0.6622	0.6467
	0.3	0.5930	0.0085	0.6061	0.5794	0.6471	0.0096	0.6660	0.6290	0.5930	0.0087	0.6062	0.5782

**Table 13:** Loss value of the surgery duration prediction system with dropout mechanism.

Architecture	Dropout	Testing dataset				Training dataset				Validation dataset			
		Mean	Std	Max	Min	Mean	Std	Max	Min	Mean	Std	Max	Min
4-256	**Without**	**0.6551**	0.0028	**0.6588**	**0.6501**	**0.6364**	0.0029	**0.6404**	**0.6312**	**0.6550**	0.0030	**0.6586**	**0.6501**
	0.1	0.6655	0.0029	0.6703	0.6605	0.6452	0.0030	0.6502	0.6408	0.6653	0.0030	0.6703	0.6613
	0.2	0.6834	**0.0014**	0.6852	0.6812	0.6662	**0.0014**	0.6682	0.6640	0.6834	**0.0010**	0.6854	0.6823
	0.3	0.6989	0.0019	0.7020	0.6956	0.6858	0.0023	0.6900	0.6811	0.6988	0.0021	0.7023	0.6953

**Table 14:** Prediction accuracy of the surgery duration prediction system with data enrichment and longer training time.

Layers	Neurons	Multiple	Epochs	Testing dataset				Training dataset				Validation dataset			
				Mean	Std	Max	Min	Mean	Std	Max	Min	Mean	Std	Max	Min
4	256	3	200	0.7711	0.0115	0.7919	0.7560	0.8468	0.0118	0.8675	0.8303	0.7714	0.0124	0.7918	0.7564
		10	200	0.8788	0.0134	0.8930	0.8453	0.8920	0.0128	0.9055	0.8602	0.8738	0.0138	0.8878	0.8398
		10	1000	**0.9485**	0.0055	0.9550	0.9402	**0.9530**	0.0046	0.9599	0.9472	**0.9473**	0.0059	0.9570	0.9389

**Table 15:** Loss value of the surgery duration prediction system with data enrichment and longer training time.

Layers	Neurons	Multiple	Epochs	Testing dataset				Training dataset				Validation dataset			
				Mean	Std	Max	Min	Mean	Std	Max	Min	Mean	Std	Max	Min
4	256	3	200	0.6551	0.0028	0.6588	0.6501	0.6364	0.0029	0.6404	0.6312	0.6550	0.0030	0.6586	0.6501
		10	200	0.6284	0.0033	0.6368	0.6248	0.6251	0.0031	0.6329	0.6218	0.6296	0.0034	0.6380	0.6262
		10	1000	**0.6110**	0.0014	0.6130	0.6093	**0.6098**	0.0011	0.6113	0.6081	**0.6112**	0.0015	0.6134	0.6088

**Table 16:** Prediction accuracy of the anesthesia emergence duration prediction system.

Layers-neurons	Testing dataset				Training dataset				Validation dataset			
	Mean	Std	Max	Min	Mean	Std	Max	Min	Mean	Std	Max	Min
3-64	0.6168	0.0137	0.6367	0.5958	0.6685	0.0156	0.6905	0.6492	0.6243	0.0133	0.6509	0.6039
3-128	0.6910	**0.0069**	0.7013	0.6812	0.7419	0.0093	0.7529	0.7240	0.6953	**0.0081**	0.7060	0.6816
3-256	0.7387	0.0085	0.7545	0.7282	0.7869	**0.0062**	0.7941	0.7743	0.7411	0.0083	0.7557	0.7266
**3-512**	**0.7391**	0.0148	0.7705	0.7241	0.7913	0.0150	0.8183	0.7758	0.7425	0.0132	0.7674	0.7266
4-64	0.6578	0.0112	0.6729	0.6372	0.7093	0.0091	0.7215	0.6921	0.6621	0.0097	0.6749	0.6437
4-128	0.7370	0.0163	0.7619	0.7180	0.7885	0.0158	0.8135	0.7652	0.7393	0.0157	0.7594	0.7124
**4-256**	**0.7836**	0.0152	**0.8131**	0.7650	0.8342	0.0132	0.8581	0.8178	0.7847	0.0157	0.8091	0.7558
4-512	0.7731	0.0181	0.7915	0.7359	0.8301	0.0167	0.8502	0.8016	0.7801	0.0177	0.8003	0.7451
5-64	0.6809	0.0153	0.7040	0.6570	0.7377	0.0150	0.7568	0.7095	0.6889	0.0187	0.7140	0.6558
5-128	0.7632	0.0201	0.7965	0.7365	0.8162	0.0207	0.8524	0.7841	0.7643	0.0201	0.7993	0.7411
**5-256**	**0.7905**	0.0158	0.8114	**0.7651**	**0.8443**	0.0151	**0.8653**	**0.8206**	**0.7924**	0.0167	**0.8117**	**0.7599**
5-512	0.7531	0.0246	0.7828	0.6956	0.8096	0.0227	0.8354	0.7561	0.7569	0.0211	0.7815	0.7060
6-64	0.6812	0.0166	0.7053	0.6477	0.7389	0.0161	0.7561	0.7023	0.6883	0.0155	0.7094	0.6537
**6-128**	**0.7454**	0.0143	0.7730	0.7210	0.8057	0.0139	0.8289	0.7780	0.7499	0.0141	0.7732	0.7225
6-256	0.7420	0.0282	0.7866	0.7030	0.8014	0.0272	0.8419	0.7649	0.7429	0.0275	0.7892	0.7029
6-512	0.7044	0.0170	0.7329	0.6812	0.7630	0.0178	0.7910	0.7351	0.7101	0.0160	0.7411	0.6905

**Table 17:** Loss value of the anesthesia emergence duration prediction system.

Layers-neurons	Testing dataset				Training dataset				Validation dataset			
	Mean	Std	Max	Min	Mean	Std	Max	Min	Mean	Std	Max	Min
3-64	0.6935	0.0033	0.6985	0.6887	0.6811	0.0038	0.6857	0.6758	0.6917	0.0032	0.6967	0.6852
3-128	0.6751	**0.0018**	0.6777	0.6726	0.6625	0.0023	0.6669	0.6598	0.6740	**0.0020**	0.6775	0.6714
3-256	0.6633	0.0021	0.6658	0.6593	0.6514	**0.0016**	0.6546	0.6495	0.6627	0.0021	0.6662	0.6590
**3-512**	**0.6632**	0.0037	0.6670	0.6554	0.6502	0.0037	0.6539	0.6435	0.6623	0.0033	0.6660	0.6561
4-64	0.6835	0.0027	0.6887	0.6801	0.6707	0.0022	0.6749	0.6676	0.6823	0.0023	0.6868	0.6792
4-128	0.6636	0.0041	0.6682	0.6573	0.6509	0.0039	0.6566	0.6448	0.6631	0.0038	0.6695	0.6584
**4-256**	**0.6520**	0.0037	**0.6566**	**0.6450**	0.6395	0.0033	0.6438	0.6337	0.6518	0.0038	0.6589	0.6459
4-512	0.6547	0.0045	0.6641	0.6501	0.6405	0.0042	0.6477	0.6355	0.6529	0.0043	0.6615	0.6481
5-64	0.6776	0.0037	0.6833	0.6721	0.6635	0.0037	0.6705	0.6588	0.6756	0.0045	0.6834	0.6695
5-128	0.6571	0.0049	0.6637	0.6490	0.6440	0.0052	0.6520	0.6350	0.6569	0.0050	0.6628	0.6482
**5-256**	**0.6503**	0.0040	0.6567	0.6450	**0.6370**	0.0037	**0.6428**	**0.6319**	**0.6499**	0.0042	**0.6578**	**0.6449**
5-512	0.6597	0.0061	0.6740	0.6525	0.6456	0.0056	0.6589	0.6393	0.6588	0.0052	0.6713	0.6526
6-64	0.6775	0.0041	0.6859	0.6717	0.6633	0.0040	0.6725	0.6590	0.6758	0.0038	0.6841	0.6703
**6-128**	**0.6616**	0.0035	0.6676	0.6550	0.6466	0.0034	0.6535	0.6409	0.6605	0.0034	0.6673	0.6548
6-256	0.6624	0.0069	0.6720	0.6514	0.6476	0.0067	0.6566	0.6376	0.6622	0.0068	0.6721	0.6508
6-512	0.6718	0.0043	0.6777	0.6646	0.6572	0.0044	0.6642	0.6503	0.6704	0.0040	0.6751	0.6629

**Table 18:** The *t*-test in 3 hidden layer architecture.

Architecture	3-128	3-256	3-512
3-64	0.0000^*∗*^	0.0000^*∗*^	0.0000^*∗*^
3-128	—	0.0000^*∗*^	0.0000^*∗*^
3-256	—	—	0.4726

**Table 19:** The *t*-test in 4 hidden layer architecture.

Architecture	4-128	4-256	4-512
4-64	0.0000^*∗*^	0.0000^*∗*^	0.0000^*∗*^
4-128	—	0.0000^*∗*^	0.0001^*∗*^
4-256	—	—	0.0892

**Table 20:** The *t*-test in 5 hidden layer architecture.

Architecture	5-128	5-256	5-512
5-64	0.0000^*∗*^	0.0000^*∗*^	0.0000^*∗*^
5-128	—	0.0017^*∗*^	0.1651
5-256	—	—	0.0004^*∗*^

**Table 21:** The *t*-test in 6 hidden layer architecture.

Architecture	6-128	6-256	6-512
6-64	0.0000^*∗*^	0.0000^*∗*^	0.0032^*∗*^
6-128	—	0.3675	0.0000^*∗*^
6-256	—	—	0.0010^*∗*^

**Table 22:** The *t*-test in 3–6 hidden layer architectures.

Architecture	4-256	5-256	6-128
3-256	0.0000^*∗*^	0.0000^*∗*^	0.1106
4-256	—	0.1680	0.0000^*∗*^
5-256	—	—	0.0000^*∗*^

**Table 23:** Running time cost of each architecture of the anesthesia emergence duration prediction system.

Neurons	Time(s)
3-64	329.91
3-128	426.52
3-256	613.93
3-512	1928.91
4-64	380.23
4-128	485.55
4-256	862.83
4-512	2709.28
5-64	399.41
5-128	579.37
5-256	1180.40
5-512	3490.63
6-64	434.80
6-128	988.21
6-256	1204.03
6-512	4245.20

**Table 24:** Prediction accuracy of the anesthesia emergence duration prediction system with dropout mechanism.

Architecture	Dropout	Testing dataset				Training dataset				Validation dataset			
		Mean	Std	Max	Min	Mean	Std	Max	Min	Mean	Std	Max	Min
4-256	**Without**	**0.7836**	0.0152	**0.8131**	**0.7650**	**0.8342**	0.0132	**0.8581**	**0.8178**	**0.7847**	0.0157	**0.8091**	**0.7558**
	0.1	0.7438	0.0114	0.7632	0.7251	0.8062	0.0135	0.8334	0.7841	0.7462	0.0144	0.7750	0.7178
	0.2	0.6582	**0.0090**	0.6773	0.6469	0.7194	**0.0079**	0.7336	0.7088	0.6680	**0.0042**	0.6743	0.6597
	0.3	0.6073	0.0105	0.6248	0.5916	0.6572	0.0117	0.6752	0.6366	0.6175	0.0087	0.6308	0.6053

**Table 25:** Loss value of the anesthesia emergence duration prediction system with dropout mechanism.

Architecture	Dropout	Testing dataset				Training dataset				Validation dataset			
		Mean	Std	Max	Min	Mean	Std	Max	Min	Mean	Std	Max	Min
4-256	**Without**	**0.6520**	0.0037	**0.6566**	**0.6450**	**0.6395**	0.0033	**0.6438**	**0.6337**	**0.6518**	0.0038	**0.6589**	**0.6459**
	0.1	0.6620	0.0028	0.6665	0.6574	0.6465	0.0033	0.6520	0.6398	0.6614	0.0036	0.6686	0.6543
	0.2	0.6832	**0.0022**	0.6860	0.6785	0.6680	**0.0019**	0.6706	0.6645	0.6807	**0.0011**	0.6826	0.6788
	0.3	0.6955	0.0026	0.6996	0.6911	0.6833	0.0028	0.6883	0.6789	0.6930	0.0021	0.6961	0.6899

**Table 26:** Prediction accuracy of the anesthesia emergence duration prediction system with data enrichment and longer training time.

Layers	Neurons	Multiple	Epochs	Testing dataset				Training dataset				Validation dataset			
				Mean	Std	Max	Min	Mean	Std	Max	Min	Mean	Std	Max	Min
4	256	3	200	0.7836	0.0152	0.8131	0.7650	0.8342	0.0132	0.8581	0.8178	0.7847	0.0157	0.8091	0.7558
		10	200	0.8956	0.0144	0.9077	0.8582	0.9056	0.0131	0.9157	0.8718	0.8954	0.0135	0.9061	0.8609
		10	1000	**0.9544**	0.0029	0.9590	0.9503	**0.9577**	0.0022	0.9610	0.9538	**0.9551**	0.0031	0.9590	0.9502

**Table 27:** Loss value of the anesthesia emergence duration prediction system with data enrichment and longer training time.

Layers	Neurons	Multiple	Epochs	Testing dataset				Training dataset				Validation dataset			
				Mean	Std	Max	Min	Mean	Std	Max	Min	Mean	Std	Max	Min
4	256	3	200	0.6520	0.0037	0.6566	0.6450	0.6395	0.0033	0.6438	0.6337	0.6518	0.0038	0.6589	0.6459
		10	200	0.6242	0.0036	0.6335	0.6212	0.6217	0.0033	0.6301	0.6192	0.6242	0.0034	0.6328	0.6216
		10	1000	**0.6095**	0.0007	0.6106	0.6084	**0.6087**	0.0005	0.6097	0.6079	**0.6094**	0.0008	0.6106	0.6084

**Table 28:** Prediction accuracy of the final combination prediction system.

Prediction system	Accuracy
The anesthesia emergence duration prediction system	0.9645
The surgery duration prediction system	0.9671
The final combination prediction system	0.9552

## Data Availability

The data used to support the findings of this study are available from the corresponding author upon request.
